# Inhibitory Effect of Seawater Pearl Hydrolysate on UVA-Induced Photoaging of Human Skin Fibroblasts

**DOI:** 10.1155/2022/1558288

**Published:** 2022-07-01

**Authors:** Siyin Han, Hongxuan Li, Fei Luo, Xin Chen, Yanhui Cen, Peng Liu, Zhenxing Chen, Taijin Lan, Jiang Lin

**Affiliations:** ^1^School of Basic Medicine, Guangxi University of Chinese Medicine, Nanning, China; ^2^The First Clinical Medical College, Guangxi University of Chinese Medicine, Nanning, China

## Abstract

This study is an investigation into the inhibitory effect of seawater pearl hydrolysate (SPH) on the UVA-induced photoaging of human skin fibroblast (HSF) cells, and the mechanism thereof. HSF cells were cultured and irradiated with a UVA 0–50 J·cm^−2^ dose gradient. The cell inhibition rate was detected using the CCK8 method, and the half-inhibitory dose was determined. Based on this, the dose of UVA irradiation for the follow-up experiment was selected to establish a photoaging model of the HSF cells. The cells were divided into a normal (N) group, UVA-irradiated (UVA) group, SPH low dose (SPHL) group, SPH medium dose (SPHM) group, and SPH high dose (SPHH) group. The photoaging model of HSF cells was established by UVA irradiation in the UVA, SPHL, SPHM, and SPHH groups; the SPHL, SPHM, and SPHH groups were treated with SPH at concentrations of 50, 100, and 200 mg·L^−1^, respectively, at the same time. After 24 and 48 h of culture, the reactive oxygen species (ROS) level of the HSF cells was detected by flow cytometry, and the required culture time of the HSF cells for the follow-up experiment was selected. The malondialdehyde and glutathione contents, as well as the activities of the superoxide dismutase, catalase, and glutathione peroxidase in the HSF cells, were detected by biochemical methods. The levels of expression of MMP-1 and collagen I protein in HSF cells were detected by the western blot test, the extent of aging of HSF cells was detected by *β*-galactosidase staining, and the apoptosis level of HSF cells was detected by flow cytometry. The results show that SPH inhibits the UVA-induced photoaging of HSF cells in a dose-dependent manner within a certain concentration range, and the effect of a concentration of 200 mg·L^–1^ was the most significant. The mechanism is related to improving the antioxidant activity of photoaging HSF cells to eliminate excessive ROS. It can inhibit apoptosis, reduce the protein expression of MMP-1, and effectively control the degradation of collagen I protein in photoaging HSF cells. Therefore, SPH offers potential for use in sunscreen cosmetics.

## 1. Introduction

Skin photoaging is often caused by environmental factors, such as ultraviolet (UV) light, smoking, and chemicals. Among these, UV exposure is the most prominent and can trigger a series of molecular and cellular reactions in the skin, resulting in rapid dynamic disorder. Human skin is composed of layers, namely, the epidermis and dermis, and the wavelength penetration of UVA exceeds that of UVB. UVA not only penetrates the epidermis and damages keratinocytes but also is absorbed by human skin fibroblasts (HSF), causing damage to the entire dermis. A large fraction of the UVA can penetrate the dermis completely and cause skin photoaging, which is manifested by skin damage, loosening, and wrinkles [1]. Skin photoaging is not merely a cosmetic problem that increases the psychological burden of patients and affects normal work and social life; it also has an etiological relationship with the occurrence of benign skin tumors, “precancerous” lesions, and skin cancer [2].

Hepu pearl, also known as seawater pearl, is an important ingredient in Chinese herbal medicine that has been used extensively for thousands of years. According to the Pharmacopoeia of the People's Republic of China, it is effective in detoxification and muscle regeneration, calming nerves, brightening eyes, and eliminating pannus formation. It is mainly used to treat palpitations, insomnia, convulsive epilepsy, red eye, pannus, nonhealing sores and ulcers, and skin spots. Li Shizhen of the Ming Dynasty believed that pearls had a beautifying effect on the skin. According to the compendium of Materia Medica, “pearls taste salty, sweet, cold, and non-toxic, calming the mind and eyes; pearls painted on the face make people moist and good color; painted on hands and feet to remove the skin; dropped phlegm, remove facial spots, detoxify acne, and make the luster white.” In the last ten years, pearl has been widely used in the treatment of skin conditions such as skin injuries, wound ulceration, bedsores, pressure ulcers, and chloasma [3–5], and its pharmacological effect on skin repair has also been studied experimentally. However, there are few reports on the prevention and treatment of skin photoaging using seawater pearls.

In the early stage, the research group selected seawater pearls for hydrolysis and obtained a series of products such as seawater pearl hydrolysate (SPH), hydrolyzed seawater pearl powder, and Zhenmi tablets and successfully developed the hydrolyzed pearl technology (national invention patents zl95106283.2, zl95108034.2, and zl95107894.1). It has been found that seawater pearl powder can prevent and treat skin photoaging in mice, and its mechanism involves the removal of excessive reactive oxygen species (ROS) from photoaging skin [6, 7]. Therefore, we studied the effect of seawater pearls on skin photoaging at the cellular level using a UVA-induced photoaging model of HSF cells to detect the ROS, oxidative damage, antioxidant level, collagen, and level of aging before and after SPH intervention on HSF cells. This study also explored the effectiveness of SPH in inhibiting the photoaging of HSF cells to provide basic research support for expanding the development and application of seawater pearls.

## 2. Materials and Methods

### 2.1. Materials

HSF cells were purchased from the Kunming Cell Bank of Typical Culture Preservation Committee of Chinese Academy of Sciences; SPH (production approval number: 450522020014) was provided by Beihai Baozhulin Marine Technology Co., Ltd.

### 2.2. Main Reagents and Instruments

Determination kits for malondialdehyde (MDA), glutathione (GSH) content, superoxide dismutase (SOD), catalase (CAT), and glutathione peroxidase (GSH-PX) were purchased from Nanjing Jiancheng Bioengineering Institute. The other suppliers are DMEM high glucose medium (HyClone); P/S antibiotic (HyClone); fetal bovine serum (Hangzhou Tianhang Biotechnology Co., Ltd.); trypsin EDTA (Jinuo Biomedical Technology Co., Ltd.); Cell Counting Kit-8 (CCK8), cell proliferation detection kit (Biosharp); reactive oxygen species (ROS) detection kit (Beyotime); Annexin V-FITC/PI apoptosis detection kit (Tianjin Sanjian Biotechnology Co., Ltd.); a UVA lamp purchased from Philips Lighting (China) Investment Co., Ltd. (the lamp power is 9W and the spectral wave is 364–366 nm); Dr-200bs enzyme labeling detector (Diatek); FACSCalibur flow meter (BD); Sco6we CO_2_ constant temperature incubator (Shell Lab); Cx-21 ordinary optical microscope (Olympus); and a Tgl-16 freezing centrifuge (Instrument of Hunan Xiangyi Laboratory).

### 2.3. Measurement of Effect of SPH on the Proliferation of HSF Cells Using the CCK8 Method

60 milliliters of 1 g·L^−1^ SPH was measured, and conventional HSF cell culture medium was added to make up the volume to 100 mL. A batch of 600 mg·L^−1^ mother liquor was prepared and sterilized through a microporous filter membrane, and conventional HSF cell culture medium was added to dilute it to 200, 100, and 50 mg·L^−1^. HSF cells were grown using a conventional medium of DMEM high glucose +10% fetal bovine serum +1% P/S antibiotics. Cells were cultured at 37°C and 5% CO_2_ in the incubator. The medium was changed every 48 h. HSF cells in a logarithmic growth phase at 1 × 10^5^ cells·ml^−1^ were digested with trypsin, prepared as a single cell suspension, added to 96-well culture plate, and cultured for 48 h. The culture medium was absorbed and discarded, cells were washed with PBS, and PBS was added to each well. The PBS was discarded, and the cells were treated with 50, 100, and 200 mg·L^−1^ SPH medium and conventional medium, respectively, for 24 and 48 h. The conventional medium was used as the control group.

### 2.4. Measurement of Effect of UVA Irradiation Dose on the Proliferation of HSF Cells Using the CCK8 Method

In the experiment, HSF cells in a logarithmic growth phase at 1 × 10^5^ cells·ml^−1^ were digested with trypsin, prepared as a single cell suspension, added to six-well plates, and cultured for 24 h. The culture medium was absorbed and discarded, cells were washed with PBS, and PBS was added to each well. The plates were irradiated under a UVA/UV lamp, and the irradiation distance was adjusted until the irradiation dose was 0/2.5/5/10/25/50 J·cm^−2^. The 0 J·cm^−2^ irradiation dose was used as the control group. After continuous culture for 24 h, some cells were transferred to a 96-well culture plate, and a 10 *μ*L CCK-8 solution was added to all the wells, followed by incubation for another 2 h in the incubator. The absorbance value at 450 nm was measured using an enzyme labeling instrument. The culture medium without cells was used as the blank group. The inhibition rate was calculated according to the formula below to determine the optimal dose of UVA irradiation. The cell inhibition rate% = (control group – experimental group)/(control group – blank group) × 100%.

### 2.5. Grouping and Administration of HSF Cells

In the experiment, HSF cells in the logarithmic growth phase were taken at 1×10^−5^cells·mL^−1^, digested with trypsin, prepared as a single cell suspension, and added to six-well plates, and cultured for 24 h. The culture medium was absorbed and discarded, the cells were washed with PBS, and PBS was added to each well. The cells were divided into five groups, namely, normal (N) group, UVA-induced group (UVA), SPH low dose group (SPHL), SPH medium dose group (SPHM), and SPH high dose group (SPHH). Except for the N group, the groups were all irradiated under a UVA/UV lamp, and the irradiation distance was adjusted until the irradiation dose was 10 J·cm^−2^. The PBS was discarded, the conventional medium was added to the N group and UVA group, and the SPHL, SPHM, and SPHH groups were treated with 50, 100, and 200 mg·L^−1^ SPH medium, respectively, for 48 h.

### 2.6. Flow Cytometry Measurement of ROS in HSF Cells

After 24 and 48 h of cell culture in six-well plates for each group, the cells were digested using trypsin, collected in 1.5 mL centrifuge tubes, and centrifuged at 300 g for 5 min, and the supernatant was removed. Serum-free medium (0.5 mL) was added to each tube, the cells were resuspended in the centrifuge tube, and 0.5 *μ*L of DCFH-DA staining solution was added. The samples were inverted and mixed several times. The cells were incubated at 37°C for 20 min and inverted to mix every 5 min. After incubation at 37°C, the samples were centrifuged at 300 g and 4°C for 3 min, the cells were precipitated, and the supernatant was removed. The cells were washed in a serum-free medium thrice, centrifuged at 300 g and 4°C for 3 min, and precipitated, and the supernatant was removed. After resuspending the cells in a serum-free medium, the cells were analyzed by flow cytometry, with excitation at 488 nm and emission at 525 nm. The level of ROS was detected, and the best detection time was determined.

### 2.7. Biochemical Detection for Contents of MDA and GSH and Activities of SOD, CAT, and GSH-PX in HSF Cells

The cells of each group were cultured for 48 h in six-well plates, digested with trypsin, collected in 1.5 mL centrifuge tubes, lysed, and centrifuged at 4°C and 2000 g for 10 min, and the supernatant was collected for analysis. Using the manufacturers' guidelines, the activities of SOD, CAT, and GSH-PX and the contents of GSH and MDA in the cells of each group were detected. The values were expressed in relative units per mg of soluble protein.

### 2.8. Western Blot Test for the Expression of MMP-1 and Collagen I Protein in HSF Cells

After culturing for 48 h in six-well plates, the cells in each group were washed twice with PBS solution, and the residual cells were dried as thoroughly as possible. An appropriate volume of total cell protein extraction reagent was added to lyse the cells for 3–5 min. The cells and reagents were placed in a 1.5 mL centrifuge tube, put in an ice bath for 30 min, and blown repeatedly with a pipette to ensure complete cell lysis. The samples were centrifuged at 13000 g and 4°C for 5 min, and the supernatant, which was the complete protein solution, was collected. A separation gel and concentrated gel were prepared, and the protein samples were placed in the sampling hole. A transfer membrane filter paper and a methanol activated PVDF membrane were prepared, and current was passed through the membrane at a constant rate of 300 mA. The transformed membrane was added to the sealing solution and sealed at room temperature for 1 h. The blocking solution was removed, and the monoclonal antibodies anti-*β*-actin, anti-MMP-1, and anti-collagen I were diluted with a suitable diluent and incubated at 4°C overnight. The diluted monoclonal antibodies were recovered and washed with TBST thrice, for 5 min each time. The diluted goat anti-rabbit IgG-HRP secondary antibody was added and incubated at room temperature for 30 min. TBST was used to wash the samples four times on a shaking table at room temperature for 5 min each time. Freshly mixed ECL solution was added to the protein side of the membrane, which was then exposed in a dark room. The film was archived, analyzed, and scanned [8].

### 2.9. Detection of Aging Level of HSF Cells by *β*-Galactosidase Staining

After 48 h of culture in six-well plates, the cells in each group were washed twice with PBS solution, and a *β*-galactosidase staining fixative was applied at room temperature for 15 min. The samples were washed three times with a PBS solution, an appropriate amount of *β*-galactosidase staining working solution was added to each hole, and the samples were incubated in a water bath at 37°C overnight. The cells were washed twice with PBS solution, and the senescence of the cells was observed under an optical microscope. The senescent cells were seen as dark blue. The average optical density of the *β*-galactosidase positive areas was measured using Image-Pro Plus software (Media Cybernetics).

### 2.10. Flow Cytometry Detection of Apoptosis Level of HSF Cells

Cells belonging to each group were cultured for 48 h in six-well plates, digested using trypsin, collected in 1.5 mL centrifuge tubes, and centrifuged at 300 g for 5 min. Following this, the supernatant was removed and 1 ml PBS was added to each tube. The cells were resuspended and centrifuged at 300 g and 4°C for 5 min, and the supernatant was discarded. The addition of 200 *μ*L precooled binding buffer resuspended the precipitated material. Annexin V-FITC (5 *μ*L) was added, and the samples were mixed well and incubated in the dark for 10 min. Then, 5 *μ*L PI was added, and the samples were mixed well and incubated in the dark for a further 5 min. Subsequently, another 200 *μ*L precooled binding buffer was added. After mixing, the extent of apoptosis in each group was detected by flow cytometry.

### 2.11. Statistical Analysis

The data are expressed as the mean ± standard error (SE), and SPSS (version 17.0) (IBM, Armonk, New York, USA) was used for statistical analysis. One-way analysis of variance (ANOVA) and the least significant difference (LSD) were used to analyze the differences between the different groups; *P* < 0.05 was considered significant. All the mathematical and statistical images were generated by Origin 8.6 software (OriginLab, Massachusetts, USA).

## 3. Results

### 3.1. Effect of SPH on the Proliferation of HSF Cells

Compared with the control group, 200 mg·L^−1^ SPH significantly improved cell proliferation rate of HSF cells after 24 h of culture (*P* < 0.05), but 50 and 100 mg·L^−1^ SPH had no significant difference after 24 h of culture (*P* > 0.05) (Figure 1). Compared with the control group, 50, 100, and 200 mg·L^−1^ SPH significantly improved cell proliferation rate of HSF cells after 48 h of culture (*P* < 0.05) (Figure 1). Thus, SPH promoted the proliferation of HSF cells without toxicity.

### 3.2. Effect of UVA Irradiation Dose on the Proliferation of HSF Cells

The cell inhibition rate increased with the increase in UVA irradiation dose, which was dose-dependent in a certain dose range. The half-inhibitory dose was 10 J·cm^−2^ (Figure 2), and 10 J·cm^−2^ was the best UVA irradiation dose for use in the follow-up experiment.

### 3.3. Effect of SPH on the ROS Level of HSF Cells

Compared with the N group, the ROS content of HSF cells in the UVA, SPHL, SPHM, and SPHH groups increased significantly after 24 and 48 h of culture (*P* < 0.05) (Figures 3(a) and 3(b)). Compared with the UVA group, the ROS content of the HSF cells in the SPHL, SPHM, and SPHH groups decreased significantly after 24 and 48 h of culture (*P* < 0.05), and the ROS content decreased as SPH increased in a dose-dependent manner within a certain concentration range (Figures 3(a) and 3(b)). Considering the stability of the experiment, 48 h was selected as the culture time for HSF cells in the follow-up experiment.

### 3.4. Effects of SPH on the Contents of MDA and GSH and SOD, CAT, and GSH-PX Activity in HSF Cells

Compared with the N group, the MDA content of HSF cells in the UVA, SPHL, SPHM, and SPHH groups increased significantly after 48 h of culture (*P* < 0.05). Compared with the UVA group, the MDA content of the HSF cells in the SPHL, SPHM, and SPHH groups decreased significantly after 48 h of culture (*P* < 0.05) (Figure 4(a)).

Compared with the N group, the content of GSH and the activities of SOD, CAT, and GSH-PX in HSF cells in the UVA and SPHL groups decreased significantly after 48 h of culture (*P*< 0.05), but there was no significant difference in the GSH content and SOD, CAT, and GSH-PX activity in the SPHM and SPHH groups (*P* > 0.05) (Figures 4(b), 4(c), 4(d), and 4(e)). Compared with the UVA group, the GSH content and SOD, CAT, and GSH-PX activities of the HSF cells in the SPHH group increased significantly after 48 h of culture (*P* < 0.05) (Figures 4(b), 4(c), 4(d), and 4(e)).

### 3.5. Effect of SPH on the Expression of MMP-1 and Collagen I Protein in HSF Cells

Compared with the N group, the relative expression of MMP-1 protein in the UVA, SPHL, and SPHM groups was significantly increased after 48 h of culture (*P* < 0.05), but there was no significant difference in the relative expression of MMP-1 protein in the SPHH group (*P* > 0.05) (Figures 5(a) and 5(b)/MMP-1). Compared with the UVA group, the relative expression of MMP-1 protein in HSF cells in the SPHL, SPHM, and SPHH groups decreased significantly after 48 h of culture (*P* < 0.05) (Figures 5(a) and 5(b)/MMP-1). The relative expression of MMP-1 protein decreased with the increase in SPH dose in a dose-dependent manner within a certain concentration range.

Compared with the N group, the relative expression of collagen I protein in HSF cells of the UVA, SPHL, SPHM, and SPHH groups decreased significantly after 48 h of culture (*P* < 0.05) (Figures 5(a) and 5(b)/collagen I). Compared with the UVA group, the relative expression of collagen I protein in HSF cells of the SPHL, SPHM, and SPHH groups increased significantly after being cultured for 48 h (*P* < 0.05) (Figures 5(a) and 5(b)/collagen I), and the relative expression of collagen I protein increased with the increase in SPH dose in a dose-dependent manner within a certain concentration range.

### 3.6. Effect of SPH on the Aging of HSF Cells

Compared with the N group, the level of aging of HSF cells in the UVA, SPHL, SPHM, and SPHH groups increased significantly after 48 h of culture (*P* < 0.05) (Figures 6(a) and 6(b)). Compared with the UVA group, the aging level of HSF cells in the SPHL, SPHM, and SPHH groups decreased significantly after 48 h of culture (*P* < 0.05) (Figures 6(a) and 6(b)), and the cell aging level decreased with the increase in the dose of SPH in a dose-dependent manner within a certain range of concentration.

### 3.7. Effect of SPH on Apoptosis of HSF Cells

Compared with the N group, the apoptosis rate of HSF cells in the UVA, SPHL, SPHM, and SPHH groups increased significantly after 48 h of culture (*P* < 0.05) (Figures 7(a) and 7(b)). Compared with the UVA group, the apoptosis rate of HSF cells in the SPHL, SPHM, and SPHH groups decreased significantly after 48 h of culture (*P* < 0.05) (Figures 7(a) and 7(b)), and the apoptosis rate decreased with the increase in the dose of SPH in a dose-dependent manner within a certain range of concentration.

## 4. Discussion

When the UV component in sunlight passes through the Earth's atmosphere, UVA and UVB in these rays can induce the production of considerable quantities of ROS in the skin [9]. The enzymatic and nonenzymatic antioxidant systems in skin cells get consumed and damaged by the excessive presence of ROS, upsetting the dynamic balance between oxidation and antioxidant systems in the body, reducing the body's ability to scavenge ROS, and increasing the accumulation of ROS in the body. Excessive ROS induces “oxidative stress,” causing oxidative damage to some cell components. The continuous accumulation of cell damage promotes changes in the cell signal transduction pathways, the role of matrix metalloproteinases (MMPs), inflammatory response, and apoptosis, resulting in apparent skin aging [10, 11]. Ancient medical books have fully affirmed the medicinal value of the “detoxification and muscle regeneration” capability of pearls. Present-day researchers have shown that pearl extract has high antioxidant capacity in vitro and in vivo and can prevent and treat diseases caused by ROS [12, 13]. Pearl extract can reduce the inflammation and apoptosis of human skin keratinocytes under UVB irradiation [14], and the aqueous extract of pearl can reduce the number of human skin fibroblasts that age under UVB irradiation [15]. Moreover, our group has carried out preliminary research and found that powdered seawater pearls can prevent and treat mouse skin photoaging, and its mechanism chiefly involves the removal of excessive ROS from photoaging skin [6, 7].

This experiment was designed to study the effectiveness and mechanism of action of SPH in inhibiting the UVA-induced photoaging of HSF cells. The photoaging model of the HSF cells was constructed by UVA irradiation. It was found that the cell inhibition rate increased with the increase in the UVA irradiation dose, and this was dose-dependent in a certain concentration range. Therefore, the half-inhibitory dose of 10 J·cm^–2^ was selected to construct the photoaging model of HSF cells. The effects of different concentrations of SPH on ROS production by the photoaging HSF cells were observed at different treatment times. After 24 and 48 h, respectively, the ROS levels in the UVA group were significantly higher than those in the N group, while the ROS levels in the SPHL, SPHM, and SPHH groups were significantly lower than those in the UVA group, showing a dose-dependent response within a certain concentration range. Considering the stability of the experiment, the subsequent studies were conducted using low, medium, and high doses of SPH to treat photoaging in HSF cells for 48 h.

Under in vivo conditions, SOD, CAT, and GSH-PX are enzymes that can remove ROS from the body, and GSH is a nonenzyme that can remove ROS, maintain the dynamic balance of oxidation and antioxidant systems, and protect skin tissue from oxidative damage [16, 17]. Excessive ROS will produce many apoptotic transcription factors and cause apoptosis [18]. It can also directly attack liposomes in skin cells and produce MDA, which causes macromolecular cross-linking reactions in skin tissue and damages dermal tissue. Chen Qiaoyun et al. reported that UVA irradiation of photoaging HSF cells can increase the ROS content and the apoptosis rate [19]. Liu Jinjuan et al. reported that the UVA irradiation of HSF cells can significantly reduce the activities of intracellular SOD and GSH-PX [20], suggesting that photoaging HSF cells undergo oxidative stress. The UVA group of photoaging HSF cells further confirmed the state of oxidative stress. After UVA irradiation, the contents of ROS and MDA and the apoptosis rate increased (*P* < 0.05), and the SOD, CAT, and GSH-PX activities and the GSH content decreased (*P* < 0.05). The SPH treatment alleviated oxidative stress and inhibited apoptosis rate by increasing the SOD, CAT, and GSH-PX activities and the GSH content of photoaging HSF cells (*P* < 0.05) and by reducing the ROS and MDA content of photoaging HSF cells (*P* < 0.05). This results in a dose-dependent effect within a certain concentration range. The effect of a concentration of 200 mg·L^–1^ was the most significant. Thus, SPH can effectively remove excess ROS and MDA, inhibit apoptosis, and enhance the ability of HSF cells to resist UVA by increasing the activities of SOD, CAT, and GSH-PX and the GSH content in photoaging HSF cells.

Collagen is the main component of the human dermis. It is mainly composed of collagen I secreted by HSF cells and plays an important role in maintaining skin fullness [21]. MMPs can promote collagen degradation, in which MMP-1 plays a major role, and collagen degradation is one of the most important reasons for the appearance of photoaging characteristics [22]. Cui reported that UVA-irradiated HSF cells produce excessive ROS, which will increase the expression of MMP-1 and MMP-3 and promote the degradation of collagen I [23]. Hseu reported that UVA-irradiated HSF cells produce excessive ROS, promoting changes in cell signal transduction pathways, increasing the expression of MMP-1, and promoting the degradation of collagen III [24]. This study found that the synthesis of MMP-1 protein in UVA-irradiated HSF cells was increased, resulting in the degradation of collagen I protein, a decrease in collagen content, and an increase in the level of cell aging. SPH can inhibit the overexpression of MMP-1 in photoaging HSF cells, increase the expression of collagen I protein, and reduce cell aging in a dose-dependent manner within a certain concentration range. The most significant concentration has been identified as 200 mg·L^−1^.

## 5. Conclusions

SPH has an inhibitory effect on UVA-induced photoaging of HSF cells, which is expressed in a dose-dependent manner within a certain concentration range. The mechanism involves improving the antioxidant activity of photoaging HSF cells to eliminate the excessive presence of ROS. SPH can inhibit apoptosis, reduce the protein expression of MMP-1, and effectively control the degradation of collagen I in photoaging HSF cells. Therefore, taking into account the excellent skin protection capabilities, SPH can be considered in the development of sunscreen cosmetics.

## Figures and Tables

**Figure 1:** Effect of SPH on the cell inhibition rate of HSF cells. ^*∗*^*P* < 0.05 versus control group; error bar = SE (*n* = 3).

**Figure 2:** Effect of UVA irradiation dose on the cell inhibition rate of HSF cells; error bar = SE (*n* = 3).

**Figure 3:** (a) Effect of SPH on ROS level of HSF cells detected by flow cytometry after 24 and 48 h. (b) Effect of SPH on ROS level of HSF cells after 24 and 48 h. ^*∗*^*P* < 0.05 versus N group; #*P* < 0.05 versus UVA group; error bar = SE (*n* = 3).

**Figure 4:** Effect of SPH on the contents of MDA (a) and GSH (b) and SOD (c), CAT (d), and GSH-PX (e) activities in HSF cells.^*∗*^*P* < 0.05 versus N group; #*P* < 0.05 versus UVA group; error bar = SE (*n* = 3).

**Figure 5:** (a) Effect of SPH on the expression of MMP-1 and collagen I protein detected by Western blot in HSF cells. (b) Semiquantitative analysis based on the relative density of MMP-1 and collagen I protein; data were normalized with *β*-actin as the internal reference. ^*∗*^*P* < 0.05 versus N group; #*P* < 0.05 versus UVA group; error bar = SE (*n* = 3).

**Figure 6:** (a) Effect of SPH on the aging level of HSF cells detected by *β*-galactosidase staining (×200), scale = 50 *μ*m. (b) Effect of SPH on the aging level of HSF cells.^*∗*^*P* < 0.05 versus N group; #*P* < 0.05 versus UVA group; error bar = SE (*n* = 3).

**Figure 7:** (a) Effect of SPH on the apoptosis level of HSF cells was detected by flow cytometry. (b) Effect of SPH on the apoptosis level of HSF cells.^*∗*^*P* < 0.05 versus N group; #*P* < 0.05 versus UVA group; error bar = SE (*n* = 3).

## Data Availability

The data used to support the findings of this study are included within the article.

## Abbreviations

SPH: Seawater pearl hydrolysate
HSF: Human skin fibroblast
UVA: Long wave ultraviolet
ROS: Reactive oxygen species
MMP-1: Matrix metalloproteinase-1
SOD: Superoxide dismutase
MDA: Malondialdehyde
GSH: Glutathione
CAT: Catalase
GSH-PX: Glutathione peroxidase.
